The article "Anti-apoptosis mechanism of triptolide based on network pharmacology in focal segmental glomerulosclerosis rats" was retracted in 2020. Reasons: results that could not be reproduced; errors in the text.

# Anti-apoptosis mechanism of triptolide based on network pharmacology in focal segmental glomerulosclerosis rats

**DOI:** 10.1042/BSR20192920

**Published:** 2020-04-28

**Authors:** Yayu Li, Xue Jiang, Litao Song, Mengdie Yang, Jing Pan

**Affiliations:** 1 Department of Nephrology, Guangxing Affiliated Hospital of Zhejiang Chinese Medical University, Hangzhou Hospital of Traditional Chinese Medicine, No. 453, Tiyuchang Road, Hangzhou City, Zhejiang Province 310007, P. R. China; 2 Department of Nephrology, Hangzhou Dingqiao Hospital, Dingqiao Branch of Hangzhou Hospital of Traditional Chinese medicine, No. 453, Tiyuchang Road, Hangzhou City, Zhejiang Province 310007, P. R. China; 3 Department of Nephrology, Zhejiang Chinese Medical University, Hangzhou, Zhejiang Province, No. 548, Binwen Road, Hangzhou City, Zhejiang Province 310000, P. R. China

**Keywords:** apoptosis, FSGS, IL4, network pharmacology, triptolide

## Abstract

Triptolide (TPL), the active component of *Tripterygium wilfordii*, exhibits anti-cancer and antioxidant functions. We aimed to explore the anti-apoptosis mechanism of TPL based on network pharmacology and *in vivo* and *in vitro* research validation using a rat model of focal segmental glomerulosclerosis (FSGS). The chemical structures and pharmacological activities of the compounds reported in *T. wilfordii* were determined and used to perform the network pharmacology analysis. The Traditional Chinese Medicine Systems Pharmacology Database (TCMSP) was then used to identify the network targets for 16 compounds from *Tripterygium wilfordii*. Our results showed that 47 overlapping genes obtained from the GeneCards and OMIM databases were involved in the occurrence and development of FSGS and used to construct the protein–protein interaction (PPI) network using the STRING database. Hub genes were identified via the MCODE plug-in of the Cytoscape software. *IL4* was the target gene of TPL in FSGS and was mainly enriched in the cell apoptosis term and p53 signaling pathway, according to Gene Ontology (GO) and Kyoto Encyclopedia of Genes and Genomes (KEGG) pathway enrichment analyses. TPL inhibited FSGS-induced cell apoptosis in rats and regulated IL4, nephrin, podocin, and p53 protein levels via using CCK8, TUNEL, and Western blot assays. The effects of IL4 overexpression, including inhibition of cell viability and promotion of apoptosis, were reversed by TPL. TPL treatment increased the expression of nephrin and podocin and decreased p53 expression in rat podocytes. In conclusion, TPL inhibited podocyte apoptosis by targeting IL4 to alleviate kidney injury in FSGS rats.

## Introduction

Focal segmental glomerulosclerosis (FSGS) is a clinical pathological syndrome, and its typical pathological feature is sclerosing lesions in the focal glomeruli and in the glomerular segment. The clinical manifestations of FSGS patients are massive proteinuria, hematuria, hypertension, and progressive decrease in renal function. The condition of 3.6% of patients with end-stage renal disease developed from FSGS [1,2]. Currently, the main clinical therapies for FSGS are immunologic drugs, glucocorticoids, and blockers of the renin–angiotensin system; however, their therapeutic effects are not satisfactory. [3]. Triptolide (TPL) is the most active and effective diterpene lactone epoxide compound isolated from Tripterygium. [4]. TPL has anti-inflammatory, anti-tumor, and immunologic effects on many diseases [4]. TPL inhibits the secretion of many cytokines, adhesion molecules, and chemokines and affects the functions of various cells, including dendritic cells and renal tubular epithelial cells [5,6]. TPL has been reported to alleviate the progression of glomerulosclerosis and the excretion rate of urinary albumin to inhibit the progression of diabetic neuropathy [6]. However, the effects and mechanisms of TPL in FSGS are still unclear. We explored the mechanism of FSGS-mediated podocyte pathogenesis based on the FSGS rat model. The present study has great significance for the diagnosis, prevention, and treatment of FSGS.

In the past, research on Chinese herbal extracts focused on a particular aspect and on finding the biological characteristics explaining the pharmacological effect with respect to this aspect [7]; however, this approach is usually one-sided. It is important to explore the relation between the acquired proof and the research results. With the development of bioinformatics and network pharmacology, proposal of a theory and proving this theory through experiments has become the main method to explore the mechanism of Chinese herb compounds [8].

Network pharmacology is based on high-throughput omics data analysis, virtual computer computing and network database retrieval, and it combines systems biology with multidirectional pharmacology [9]. The mechanism of drug action was researched via the construction and analysis of biological networks. The systematic and holistic nature of network pharmacology is consistent with the characteristics of Chinese herbs, which exhibit multi-components, multi-targets, and systematic regulation. It has been widely used to explore the pharmacological basis of Chinese medicine and the drug mechanism and to interpret drug compatibility [10,11]. Network pharmacology has been recognized by many Chinese medicine researchers [12]. The multi-component and multi-target network research mode breaks the traditional research mode of a single ingredient and a single target, providing a new method for comprehensive analysis of the mechanism of the compounds [13]. In the early stage, a total of 47 target genes and the corresponding 16 active constituents of Tripterygium were used to construct the ingredient-target network. The present study mainly explores the mechanism of TPL in FSGS through bioinformatics and functional experiments.

## Materials and methods

### Construction of the potential compound database for tripterygium

Using the Traditional Chinese Medicine Systems Pharmacology Database and Analysis Platform (http://lsp.nwu.edu.cn/tcmsp.php, TCMSP), each candidate’s drug ability was analyzed according to its oral bioavailability (OB) and drug-likeness (DL) indices recommended by the TCMSP. OB refers to the degree and rate of drug absorption into the circulatory system, which is an important indicator for objectively evaluating the intrinsic quality of drugs. The higher the OB of the compound, the more likely it is to be developed for clinical application. DL is the sum of the pharmacokinetic properties and safety, which arises from the interactions among the physicochemical properties and structural factors, including solubility, permeability, and stability. It can be used to optimize compounds, analyze the results of drug activity, predict *in vivo* pharmacokinetics, direct structure modifications, etc. As the TCMSP recommends, molecules with OB ≥ 30% and DL ≥ 0.18 were considered to exhibit relatively better pharmacological properties and were screened out as candidate compounds for further analysis.

### Construction of the disease–target–compound network

To comprehensively understand the molecular mechanisms, disease–compound–target networks were constructed using the Cytoscape visualization software 3.7.1. All target genes related to FSGC were obtained from the GeneCards database (https://www.genecards.org/). All the candidate compounds of Tripterygium were retrieved from the TCMSP to obtain the associated targets. Next, disease, compounds, and targets were inputted into the software, and a disease–compound–target interaction network was constructed. In the process of constructing the network, the layout algorithm (attribute circle layout) was applied. We can set the geometric position of every node and visually display the network topology using color, graphics, and symbols, making reasonable arrangements for every node and creating a clear visual effect. Degree and betweenness centrality are two important parameters of the topology structure, which were used to evaluate the essentiality of each target and compound.

### PPI network construction and module analysis

Search Tool for the Retrieval of Interacting Genes (STRING, https://string-db.org) is an online tool and used to construct the PPI network with confidence network edges and a medium confidence of 0.400 as the product criteria. Cytoscape 7.1.0 was used to perform the visualization of PPI network. The Molecular Complex Detection (MCODE) plug-in was used to screen the significant modules in the PPI network with a degree cut-off = 2, node score cut-off = 0.2, k-core = 2, and maximum depth = 100. The corresponding proteins in the central nodes and highly degree were potential core proteins encoded by key candidate genes that have important physiological regulatory functions.

### GO terms and KEGG pathway enrichment analysis

The Database for Annotation, Visualization, and Integrated Discovery (DAVID) database was used to perform GO enrichment analysis and KEGG pathway enrichment analysis. The GO terms were classified into three categories: biological process (BP), cellular component (CC); and molecular function (MF). *P*<0.01 was considered to indicate a statistically significant difference.

### Animals

A total of 40 Sprague Dawley (SD) rats (male, weighing 160–180 g) were provided by Yison Bio co.LTD (Shanghai, China). Animals were housed individually in polycarbonate cages with wood chip bedding and were maintained in an air-conditioned animal room (temperature: 24°C, relative humidity: 55 ± 5%) on a 12-h light/dark cycle. Each animal experiment was carried out following the local Care for Laboratory Animals guidelines formulated by the Animal Experimental Center. The Ethics Committee had approved the studies using laboratory animals at the Guangxing Affiliated Hospital of Zhejiang Chinese Medical University.

### FSGS model establishment

All rats were randomly divided into a sham operation group (Sham), model group (FSGS), a group administered 80 mg/(kg·d) of Tripterygium by gavage (TPL(80)+FSGS), and a group administered 160 mg/(kg · d) of Tripterygium by gavage (TPL(160)+FSGS) (*n*=10 rats/group). One day before the operation, the TPL (80 or 160)+FSGS groups were administered TPL (Purifa Technology Development Co. Ltd., Chengdu, Sichuan, China) 80 or 160 mg/(kg d) by gavage; the Sham and FSGS groups were given isovolumic normal saline till the end of the experiment. The animals were intraperitoneally anesthetized with pentobarbital sodium (60 mg/kg body weight) and then placed on a homeothermic pad to maintain a core body temperature of 37°C to establish the FSGS model. The rats were first subjected to unilateral nephrectomy (left side) on day 1 and then injected in the caudal vein with adriamycin 5 mg/kg (on day 7) and adriamycin 3 mg/kg (on day 28) dissolved in 0.9% saline at a dilution of 2 mg/ml. Meanwhile, the kidneys of the control rats were exposed without dissecting the kidney tissue, followed by layer-by-layer suturing. These rats were then injected with saline on days 7 and 28 through the tail vein after the sham operation. Eight weeks post-surgery, blood samples were obtained from the tail veins, and the animals were killed. Following adequate anesthesia with pentobarbital sodium (180 mg/kg body weight), the organs were removed, frozen, or fixed in 4% paraformaldehyde. The serum and whole kidneys were harvested for biochemical, histological, and molecular analyses. The urinary protein levels of the rats were quantified before the end of the experiment. Animals with >100 mg/24 h urinary protein indicated successful establishment of the model, and they were included in subsequent experiments.

### Histological analyses

The kidney tissues were fixed with 4% paraformaldehyde and embedded in paraffin. For histological analysis of lesions, 3 μm thick tissue sections were deparaffinized and stained with hematoxylin and eosin (HE) and periodic acid–Schiff (PAS). To calculate the degree of focal glomerular sclerosis, 40–60 glomeruli from each stained specimen were examined. The degree of sclerosis in each glomerulus was subjectively graded on a scale of 0–4 as follows: Grade 0, no change; Grade 1, sclerotic area less than or equal to 25% of the glomerulus or the presence of distinct adhesion between the capillary tuft and Bowman’s capsule; Grade 2, sclerosis of 25–50% of the total glomerular area; Grade 3, sclerosis of 50–75% of the total glomerular area; and Grade 4, sclerosis of more than 75% of the glomerulus. The glomerular sclerosis index (GSI) was calculated using the following formula:

GSI=(1×N1)+(2×N2)+(3×N3)+(4×N4)/(N0+N1+N2+N3+N4)

where *N* is the number of glomeruli for each grade of sclerosis.

### Terminal dUTP nick-end labeling (TUNEL) staining

An apoptosis detection kit (Promega, Madison, WI) was used to detect apoptosis according to a previously described method [14]. In brief, renal sections were subjected to TUNEL staining in accordance with the manufacturer’s instructions. Later, IF microscopy was used to analyze the samples using a Zeiss Axiovert 200 M fluorescent microscope equipped with an AxioCamMR3 camera. Six fields (magnification 400×) were randomly selected from every section from 10 different rats, and cells with positive TUNEL staining were analyzed.

### Glucose treatment and cell culture

Rat glomerular podocytes were provided by Yubo Bio-Technique Co. Ltd (Shanghai, China), which were then cultivated according to a previously described method. Rat podocytes were cultivated in RPMI 1640 (Sigma-Aldrich, U.S.A.) containing streptomycin (100 μg/ml), penicillin (100 U/ml) (Solarbio, Beijing, China), and 10% fetal bovine serum (FBS, Gibco, NY, Grand Island). Subsequently, the cells were cultivated in a 5% CO_2_ incubator (Heraeus, Japan) at 33°C with interferon-γ (IFN-γ, 40 units/ml, Sigma, St Louis, MO, U.S.A.). Later, to induce differentiation, the podocytes were maintained at 37°C for 2 weeks in the absence of interferon. Podocytes (3 × 10^5^ cells/ml) were plated into 6-well plates in the presence of complete medium. After 24 h of standing, the podocytes were subjected to 24 and 48 h of TPL treatment at different concentrations (0, 5, 10, 20, 40, and 80 µmol/ml) before they were collected for subsequent analysis.

### Transient transfection of plasmid DNA or siRNA

The previously described human IL4 plasmid DNA at full length [15] was utilized to increase IL4 expression in cells via using transient transfection. pcDNA3.1-Myc/His EV plasmid (Life technologies) and On-Target Plus scramble RNA (Dharmacon) were used as transient transfection controls. Sequences for IL4 overexpression was ACAUUACUGCCUGAAGGGUGAAUUAACGC.

### Counting Kit-8 (CCK-8) assay

Cells were grown into the 96-well plates at the density of 1 × 10^5^ cells/well, followed by 24 and 48 h of culture. Afterwards, cell viability was detected via using the CCK-8 kit (Dojindo Molecular Technologies, Gaithersburg, MD, U.S.A.). Then, cells in each group were cultivated for additional 24 and 48 h, respectively. Next, the CCK8 solution (10 μl) was added into cell at 37°C for 4 h. The absorbance was determined at 450 nm for obtaining the cell growth curve by the iMark microplate absorbance reader (Bio-Rad Laboratories, Inc., Hercules, CA, U.S.A.). Each experiment was carried out in triplicate.

### Apoptosis detected by flow cytometry using Annexin V-FITC/PI staining

Cell apoptosis was examined using the Annexin V-FITC/PI kit. Briefly, the cells were subjected to 0.25% trypsin digestion (Thermo Fisher Scientific, Waltham, MA, U.S.A.), followed by two washes with cold PBS; resuspension with 5 μl of PI, 5 μl of annexin V-FITC, and 500 μl of binding buffer; and incubation under 15 min of ambient temperature in the dark. Typically, Annexin V-FITC can bind to phosphatidylserine located on the outer apoptotic cell membrane, whereas PI can penetrate and stain cells with impaired membranes before binding to and labeling DNA. Data were collected using a flow cytometer (BD FACSCalibur; BD Biosciences, Franklin Lakes, NJ, U.S.A.) and analyzed by FlowJo. Clumped cells were excluded from the FSC-H/FSC-A dot plot for selecting the single cells. Cells in the annexin V-FITC-/PI+, annexin V-FITC+/PI+, and annexin V-FITC+/PI− quadrants were regarded as apoptotic cells.

### Western blotting

Cells were subjected to lysis within the RIPA buffer (Beyotime, Shanghai, China) to collect the lysates in tubes, followed by 20 min of centrifugation at 4°C at 12,000 ***g***. Later, all supernatants were extracted, and protein content was measured by the BCA Protein Quantitative Kit (Beyotime, Shanghai, China). Then, Western blotting had been carried out in accordance with the instruction. Afterwards, 20 μg protein was subjected to 10% SDS-PAGE for separation, followed by transfer onto the PVDF membranes (Millipore, Billerica, MA, U.S.A.). Later, the membranes were blocked using 5% skimmed milk for 1 h, followed by overnight incubation with anti-IL-4 (dilution 1:8000, Abcam, Cambridge, MA, U.S.A., ab69811), nephrin (Abcam, ab227806; diluted at 1:1200), podocin (Abcam, ab50339; diluted at 1:1000), phosph (p)-Stat6 (BioVision, U.S.A., 3476-100; diluted at 1:1000), and GAPDH (Abcam, Cambridge, MA, U.S.A., ab181602; dilution 1:1000) rabbit anti-human antibodies, at 4°C, separately. Afterwards, cells were subjected to 1 h incubation with HRP-labeled secondary antibody (goat anti-rabbit antibody, Abcam, Cambridge, MA, U.S.A., ab116282; dilution 1:2000), prior to ECL detection. The Immobilon Western Chemiluminescent kit (WBKLS0100; Millipore, U.S.A.) was used to reveal the reactive bands using Roche Cobas e601 automated chemiluminescence image analysis system (Roche, U.S.A.).

### Reverse transcription-quantitative polymerase chain reaction (RT-qPCR) assay

The GAPDH and IL-4 mRNA expression was detected through RT-qPCR. Total cellular RNA was isolated by TRIzol (Invitrogen, Carlsbad, CA, U.S.A.) in accordance with manufacturer protocols. Afterwards, cDNA was synthesized by reverse transcription of RNA according to the reactions below: RNase-free dH2O, total RNA (500 ng), and 5×PrimeScript RT Master Mix (2 μl) were added until the final volume became 10 μl. The Prism 7500 (ABI, Foster City, CA, U.S.A.) was employed for real-time PCR following the standard protocol of SYBR green assay. Primers used in the present study were shown below: IL-4-F: 5′-GATCACAAAGTACTGGTCCTGG-3′. Notably, GAPDH served as a normal control, with the primers of 5′-CACCCTGTTGCTGTAGCCAAA-3′ (reverse) and 5′-TGACTTCAACAGCGACACCCA-3′ (forward). Later, qPCR was carried out in triplicate using 7500 Real-Time PCR ABI system (ABI, U.S.A.) at a format of the 96-well plate. The reaction volume of 20 μl was prepared for PCR, which included forward primer (0.8 μl, 10 μM), RNase-free dH2O (7.4 μl),reverse primer (0.8 μl, 10 μM), 2×FastStart Universal SYBR Green Master (10 μl, ROX; Invitrogen, Guangzhou, China), and cDNA (1 μl). Besides, the PCR conditions were as follows, 10 min at 95°C, followed by 15 s at 95°C for 40 cycles, and 1 min at 60°C. The sequence detection software (1.6.3, Applied Biosystems, ABI, U.S.A.) was used for data analysis. Relative GAPDH or IL-4 mRNA level was measured and standardized according to 2^−ΔΔCt^ method based on GAPDH.

### Statistical analyses

SPSS 15.0 (http://spss.en.softonic.com/) was employed for all statistical analyses. Differences between two groups were analyzed through independent sample *t*-test, whereas those among several groups were examined by one-way analysis of variance (ANOVA). Rate was compared by chi-square test. The statistically significant level was set as *P*<0.01 or *P*<0.05.

## Results

### Identification of active compounds in *Tripterygium wilfordii*

Using TCMSP databases (http://lsp.nwsuaf.edu.cn/tcmsp.php), 144 compounds of Tripterygium were retrieved. According to the criteria of DL ≥ 0.18 and OB ≥ 30%, a total of 51 chemical ingredients were selected (Table 1). TPL was verified as an active ingredient of *T. wilfordii*.

**Table 1:** Information for 51 chemical ingredients of tripterygium

Mol ID	Molecule name	OB (%)	DL
MOL000211	Mairin	55.38	0.78
MOL000296	Hederagenin	36.91	0.75
MOL000358	Beta-sitosterol	36.91	0.75
MOL000422	Kaempferol	41.88	0.24
MOL000449	Stigmasterol	43.83	0.76
MOL002058	40957-99-1	57.2	0.62
MOL003182	(+)-Medioresinol di-O-beta-D-glucopyranoside_qt	60.69	0.62
MOL003184	81827-74-9	45.42	0.53
MOL003185	(1R,4aR,10aS)-5-hydroxy-1-(hydroxymethyl)-7-isopropyl-8-methoxy-1,4a -dimethyl-4,9,10,10a-tetrahydro-3H-phenanthren-2-one	48.84	0.38
MOL003187	Triptolide	51.29	0.68
MOL003188	Tripchlorolide	78.72	0.72
MOL003189	WILFORLIDE A	35.66	0.72
MOL003192	Triptonide	67.66	0.7
MOL003196	Tryptophenolide	48.5	0.44
MOL003198	5 alpha-Benzoyl-4 alpha-hydroxy-1 beta,8 alpha-dinicotinoyl-dihydro-agarofuran	35.26	0.72
MOL003199	5,8-Dihydroxy-7-(4-hydroxy-5-methyl-coumarin-3)-coumarin	61.85	0.54
MOL003206	Canin	77.41	0.33
MOL003208	Celafurine	72.94	0.44
MOL003209	Celallocinnine	83.47	0.59
MOL003210	Celapanine	30.18	0.82
MOL003211	Celaxanthin	47.37	0.58
MOL003217	Isoxanthohumol	56.81	0.39
MOL003222	Salazinic acid	36.34	0.76
MOL003224	Tripdiotolnide	56.4	0.67
MOL003225	Hypodiolide A	76.13	0.49
MOL003229	Triptinin B	34.73	0.32
MOL003231	Triptoditerpenic acid B	40.02	0.36
MOL003232	Triptofordin B1	39.55	0.84
MOL003233	Triptofordin B2	107.71	0.76
MOL003234	Triptofordin C2	30.16	0.76
MOL003235	Triptofordin D1	32	0.75
MOL003236	Triptofordin D2	30.38	0.69
MOL003238	Triptofordin F1	33.91	0.6
MOL003239	Triptofordin F2	33.62	0.67
MOL003241	Triptofordin F4	31.37	0.67
MOL003242	Triptofordinine A2	30.78	0.47
MOL003244	Triptonide	68.45	0.68
MOL003245	Triptonoditerpenic acid	42.56	0.39
MOL003248	Triptonoterpene	48.57	0.28
MOL003266	21-Hydroxy-30-norhopan-22-one	34.11	0.77
MOL003267	Wilformine	46.32	0.2
MOL003278	Salaspermic acid	32.19	0.63
MOL003279	99694-86-7	75.23	0.66
MOL003280	TRIPTONOLIDE	49.51	0.49
MOL003283	(2R,3R,4S)-4-(4-hydroxy-3-methoxy-phenyl)-7-methoxy-2,3-dimethylol-tetralin-6-ol	66.51	0.39
MOL004443	Zhebeiresinol	58.72	0.19
MOL005828	Nobiletin	61.67	0.52
MOL007415	[(2S)-2-[[(2S)-2-(benzoylamino)-3-phenylpropanoyl]amino]-3-phenylpropyl] acetate	58.02	0.52
MOL007535	(5S,8S,9S,10R,13R,14S,17R)-17-[(1R,4R)-4-ethyl-1,5-dimethylhexyl] -10,13-dimethyl-2,4,5,7,8,9,11,12,14,15,16, 17-dodecahydro-1H-cyclopenta [a]phenanthrene-3,6-dione	33.12	0.79
MOL009386	3,3′-bis-(3,4-dihydro-4-hydroxy-6-methoxy)-2H-1-benzopyran	52.11	0.54
MOL011169	Peroxyergosterol	44.39	0.82

### Construction of the disease–target–compound network and PPI network

The TCMSP and GeneCards databases were used to predict the potential targets for each compound in FSGS. As a result, 123 target genes from the GeneCards database were verified to be involved in FSGS (Table 2), and 695 target genes of Tripterygium from the TCMSP database were verified (Table 3). After importing data into Cytoscape, a disease–compound–target network was constructed (Figure 1A). In addition, 47 overlapping target genes from two databases (TCMSP and GeneCards) were used to construct the PPI network. *IL4* obtained from the most significant module of the PPI network was verified as a key by using the MCODE plug-in of Cytoscape software, and it was found to be involved in FSGS (Figure 1B–D).

**Figure 1:** Disease–Compound–Target network and PPI network (**A**) The triptergium-target network of FSGS. (**B**) 47 overlapped target genes were from two databases (TCMSP and GeneCards). (**C**) 47 overlapped target genes were used to constructed PPI network and hub genes in PPI network. (**D**) Module and key gene were analysis and screened by using the MCODE plug-in Cytoscape software.

**Table 2:** Information for target genes of FSGS from GeneCards database

Gene symbol	Description
INF2	Inverted Formin, FH2 And WH2 Domain Containing
TRPC6	Transient Receptor Potential Cation Channel Subfamily C Member 6
CD2AP	CD2 Associated Protein
ACTN4	Actinin Alpha 4
NPHS1	NPHS1, Nephrin
NPHS2	NPHS2, Podocin
PAX2	Paired Box 2
WT1	Wilms Tumor 1
CRB2	Crumbs 2, Cell Polarity Complex Component
MYO1E	Myosin IE
APOL1	Apolipoprotein L1
ANLN	Anillin Actin Binding Protein
PLCE1	Phospholipase C Epsilon 1
PTPRO	Protein Tyrosine Phosphatase, Receptor Type O
NUP107	Nucleoporin 107
ARHGAP24	Rho GTPase Activating Protein 24
SMARCAL1	SWI/SNF Related, Matrix Associated, Actin Dependent Regulator Of Chromatin, Subfamily A Like 1
COQ6	Coenzyme Q6, Monooxygenase
LAMB2	Laminin Subunit Beta 2
COL4A3	Collagen Type IV Alpha 3 Chain
NUP93	Nucleoporin 93
COQ8B	Coenzyme Q8B
SYNPO	Synaptopodin
TGFB1	Transforming Growth Factor Beta 1
CLCN5	Chloride Voltage-Gated Channel 5
MYH9	Myosin Heavy Chain 9
LOC107985291	Uncharacterized LOC107985291
COL4A4	Collagen Type IV Alpha 4 Chain
SGPL1	Sphingosine-1-Phosphate Lyase 1
NUP205	Nucleoporin 205
PLAUR	Plasminogen Activator, Urokinase Receptor
ACE	Angiotensin I Converting Enzyme
COL4A5	Collagen Type IV Alpha 5 Chain
CDKN1C	Cyclin Dependent Kinase Inhibitor 1C
KIRREL2	Kirre Like Nephrin Family Adhesion Molecule 2
CDKN1A	Cyclin Dependent Kinase Inhibitor 1A
EMP2	Epithelial Membrane Protein 2
CDKN1B	Cyclin Dependent Kinase Inhibitor 1B
ILK	Integrin Linked Kinase
CD80	CD80 Molecule
SLC37A4	Solute Carrier Family 37 Member 4
CTNNB1	Catenin Beta 1
ITGA3	Integrin Subunit Alpha 3
SCARB2	Scavenger Receptor Class B Member 2
AGRN	Agrin
ALG1	ALG1, Chitobiosyldiphosphodolichol Beta-Mannosyltransferase
PLEKHH2	Pleckstrin Homology, MyTH4 And FERM Domain Containing H2
MPV17	Mitochondrial Inner Membrane Protein MPV17
ALB	Albumin
WDR73	WD Repeat Domain 73
REN	Renin
NARS2	Asparaginyl-TRNA Synthetase 2, Mitochondrial
SEC61A1	Sec61 Translocon Alpha 1 Subunit
ZNF592	Zinc Finger Protein 592
ITGB4	Integrin Subunit Beta 4
IL1B	Interleukin 1 Beta
OSGEP	O-Sialoglycoprotein Endopeptidase
TP53RK	TP53 Regulating Kinase
TPRKB	TP53RK Binding Protein
LAGE3	L Antigen Family Member 3
G6PC	Glucose-6-Phosphatase Catalytic Subunit
VPS33A	VPS33A, CORVET/HOPS Core Subunit
LPL	Lipoprotein Lipase
ICAM1	Intercellular Adhesion Molecule 1
CDH17	Cadherin 17
MAGI2	Membrane Associated Guanylate Kinase, WW And PDZ Domain Containing 2
ARHGDIA	Rho GDP Dissociation Inhibitor Alpha
DNAI1	Dynein Axonemal Intermediate Chain 1
ANKFY1	Ankyrin Repeat And FYVE Domain Containing 1
BSND	Barttin CLCNK Type Accessory Beta Subunit
MAX	MYC Associated Factor X
FAH	Fumarylacetoacetate Hydrolase
VHL	Von Hippel–Lindau Tumor Suppressor
LYZ	Lysozyme
AFP	Alpha Fetoprotein
RET	Ret Proto-Oncogene
MDH2	Malate Dehydrogenase 2
SDHB	Succinate Dehydrogenase Complex Iron Sulfur Subunit B
SDHA	Succinate Dehydrogenase Complex Flavoprotein Subunit A
MUC1	Mucin 1, Cell Surface Associated
FH	Fumarate Hydratase
KIF1B	Kinesin Family Member 1B
SDHC	Succinate Dehydrogenase Complex Subunit C
SDHD	Succinate Dehydrogenase Complex Subunit D
COQ2	Coenzyme Q2, Polyprenyltransferase
PLEC	Plectin
SDHAF2	Succinate Dehydrogenase Complex Assembly Factor 2
TMEM127	Transmembrane Protein 127
ELP1	Elongator Complex Protein 1
ACHE	Acetylcholinesterase (Cartwright Blood Group)
TJP1	Tight Junction Protein 1
KIRREL1	Kirre Like Nephrin Family Adhesion Molecule 1
NEDE	Nephropathy, Progressive, With Deafness
PDGFA	Platelet Derived Growth Factor Subunit A
CD40LG	CD40 Ligand
ENTPD5	Ectonucleoside Triphosphate Diphosphohydrolase 5
GAPVD1	GTPase Activating Protein And VPS9 Domains 1
NUMBL	NUMB Like, Endocytic Adaptor Protein
KANK2	KN Motif And Ankyrin Repeat Domains 2
CD79A	CD79a Molecule
BRAF	B-Raf Proto-Oncogene, Serine/Threonine Kinase
NDN	Necdin, MAGE Family Member
AXDND1	Axonemal Dynein Light Chain Domain Containing 1
PLCE1-AS1	PLCE1 Antisense RNA 1
LMX1B	LIM Homeobox Transcription Factor 1 Beta
WT1-AS	WT1 Antisense RNA
PODXL	Podocalyxin Like
INS	Insulin
VIM	Vimentin
NAGLU	N-Acetyl-Alpha-Glucosaminidase
ACTB	Actin Beta
NR5A1	Nuclear Receptor Subfamily 5 Group A Member 1
LOC105369403	Uncharacterized LOC105369403
ITGB1	Integrin Subunit Beta 1
UTRN	Utrophin
ALG13	ALG13, UDP-N-Acetylglucosaminyltransferase Subunit
CLDN1	Claudin 1
CCN2	Cellular Communication Network Factor 2
OCRL	OCRL, Inositol Polyphosphate-5-Phosphatase
CMIP	C-Maf Inducing Protein
ACTL7B	Actin Like 7B
NXF5	Nuclear RNA Export Factor 5
CUBN	Cubilin
LCAT	Lecithin-Cholesterol Acyltransferase
AGTR1	Angiotensin II Receptor Type 1
LRP2	LDL Receptor Related Protein 2
TNF	Tumor Necrosis Factor
BAX	BCL2 Associated X, Apoptosis Regulator
TLR4	Toll Like Receptor 4
ITGB3	Integrin Subunit Beta 3
DAG1	Dystroglycan 1
CCL2	C-C Motif Chemokine Ligand 2
NGF	Nerve Growth Factor
CYCS	Cytochrome *C*, Somatic
VTN	Vitronectin
SMAD3	SMAD Family Member 3
NOTCH1	Notch 1
WNT1	Wnt Family Member 1
CCNA2	Cyclin A2
NTRK2	Neurotrophic Receptor Tyrosine Kinase 2
DBH	Dopamine Beta-Hydroxylase
SMARCA4	SWI/SNF Related, Matrix Associated, Actin Dependent Regulator Of Chromatin, Subfamily A, Member 4
SMARCA2	SWI/SNF Related, Matrix Associated, Actin Dependent Regulator Of Chromatin, Subfamily A, Member 2
IDS	Iduronate 2-Sulfatase
PYGL	Glycogen Phosphorylase L
GUSB	Glucuronidase Beta
GALK1	Galactokinase 1
APRT	Adenine Phosphoribosyltransferase
ALAD	Aminolevulinate Dehydratase
PAX6	Paired Box 6
SOX9	SRY-Box 9
CLCN7	Chloride Voltage-Gated Channel 7
ALDOB	Aldolase, Fructose-Bisphosphate B
HYAL1	Hyaluronidase 1
PHKA2	Phosphorylase Kinase Regulatory Subunit Alpha 2
HEXA	Hexosaminidase Subunit Alpha
HPD	4-Hydroxyphenylpyruvate Dioxygenase
ARSB	Arylsulfatase B
APOC2	Apolipoprotein C2
GALNS	Galactosamine (N-Acetyl)-6-Sulfatase
CLCNKB	Chloride Voltage-Gated Channel Kb
AMH	Anti-Mullerian Hormone
GNS	Glucosamine (N-Acetyl)-6-Sulfatase
SGSH	N-Sulfoglucosamine Sulfohydrolase
FGF9	Fibroblast Growth Factor 9
CLCN4	Chloride Voltage-Gated Channel 4
IDUA	Iduronidase, Alpha-L-
TIA1	TIA1 Cytotoxic Granule Associated RNA Binding Protein
INPP5B	Inositol Polyphosphate-5-Phosphatase B
CLCNKA	Chloride Voltage-Gated Channel Ka
CLDN16	Claudin 16
G6PC3	Glucose-6-Phosphatase Catalytic Subunit 3
BAZ1A	Bromodomain Adjacent To Zinc Finger Domain 1A
GSTZ1	Glutathione S-Transferase Zeta 1
CIAO1	Cytosolic Iron-Sulfur Assembly Component 1
ELP3	Elongator Acetyltransferase Complex Subunit 3
SMARCA1	SWI/SNF Related, Matrix Associated, Actin Dependent Regulator Of Chromatin, Subfamily A, Member 1
GABRE	Gamma-Aminobutyric Acid Type A Receptor Epsilon Subunit
USP19	Ubiquitin Specific Peptidase 19
ELP2	Elongator Acetyltransferase Complex Subunit 2
TIMM8B	Translocase Of Inner Mitochondrial Membrane 8 Homolog B
CPSF7	Cleavage And Polyadenylation Specific Factor 7
ASTN1	Astrotactin 1
LHX9	LIM Homeobox 9
SRY	Sex Determining Region Y
ZNF274	Zinc Finger Protein 274
ARSH	Arylsulfatase Family Member H
MFRP	Membrane Frizzled-Related Protein
TECPR2	Tectonin Beta-Propeller Repeat Containing 2
YIPF3	Yip1 Domain Family Member 3
ZFY	Zinc Finger Protein Y-Linked
FAM47E	Family With Sequence Similarity 47 Member E
LOC100506321	Uncharacterized LOC100506321
LAMB1	Laminin Subunit Beta 1
PCNA	Proliferating Cell Nuclear Antigen
MT-ND2	Mitochondrially Encoded NADH:Ubiquinone Oxidoreductase Core Subunit 2
MT-CO1	Mitochondrially Encoded Cytochrome C Oxidase I
MT-CO2	Mitochondrially Encoded Cytochrome C Oxidase II
CTSL	Cathepsin L
SERPINE1	Serpin Family E Member 1
EZR	Ezrin
IFI27	Interferon Alpha Inducible Protein 27
AKT1	AKT Serine/Threonine Kinase 1
CCND1	Cyclin D1
BMP6	Bone Morphogenetic Protein 6
LMNA	Lamin A/C
CR1	Complement C3b/C4b Receptor 1 (Knops Blood Group)
SMAD2	SMAD Family Member 2
AGT	Angiotensinogen
CLU	Clusterin
CCNB1	Cyclin B1
PPARG	Peroxisome Proliferator Activated Receptor Gamma
TIMP2	TIMP Metallopeptidase Inhibitor 2
IL6	Interleukin 6
EDN1	Endothelin 1
DNM1	Dynamin 1
CDH2	Cadherin 2
JAG1	Jagged 1
MME	Membrane Metalloendopeptidase
CAMK2B	Calcium/Calmodulin Dependent Protein Kinase II Beta
FYN	FYN Proto-Oncogene, Src Family Tyrosine Kinase
LRP5	LDL Receptor Related Protein 5
PTK2	Protein Tyrosine Kinase 2
LRP6	LDL Receptor Related Protein 6
VCL	Vinculin
ITGAV	Integrin Subunit Alpha V
KRT8	Keratin 8
PLCG1	Phospholipase C Gamma 1
DKK1	Dickkopf WNT Signaling Pathway Inhibitor 1
CD151	CD151 Molecule (Raph Blood Group)
NCK1	NCK Adaptor Protein 1
YWHAQ	Tyrosine 3-Monooxygenase/Tryptophan 5-Monooxygenase Activation Protein Theta
IRF6	Interferon Regulatory Factor 6
PARVA	Parvin Alpha
KIRREL3	Kirre Like Nephrin Family Adhesion Molecule 3
MKI67	Marker Of Proliferation Ki-67
LAMA5	Laminin Subunit Alpha 5
TLN1	Talin 1
LIMS1	LIM Zinc Finger Domain Containing 1
FAT1	FAT Atypical Cadherin 1
MIR4758	MicroRNA 4758
MIR6852	MicroRNA 6852
IL2	Interleukin 2
PON1	Paraoxonase 1
FN1	Fibronectin 1
IL2RA	Interleukin 2 Receptor Subunit Alpha
IL10	Interleukin 10
NOS2	Nitric Oxide Synthase 2
CABIN1	Calcineurin Binding Protein 1
FGF2	Fibroblast Growth Factor 2
LCN2	Lipocalin 2
LAMC1	Laminin Subunit Gamma 1
CDK2	Cyclin Dependent Kinase 2
APOE	Apolipoprotein E
PLA2G7	Phospholipase A2 Group VII
HIF1A	Hypoxia Inducible Factor 1 Subunit Alpha
PAFAH1B1	Platelet Activating Factor Acetylhydrolase 1b Regulatory Subunit 1
F2R	Coagulation Factor II Thrombin Receptor
GNA12	G Protein Subunit Alpha 12
TTR	Transthyretin
MMP14	Matrix Metallopeptidase 14
ACTN1	Actinin Alpha 1
ATP7A	ATPase Copper Transporting Alpha
IGFBP3	Insulin Like Growth Factor Binding Protein 3
ATP6AP2	ATPase H+ Transporting Accessory Protein 2
GNE	Glucosamine (UDP-N-Acetyl)-2-Epimerase/N-Acetylmannosamine Kinase
S100A4	S100 Calcium Binding Protein A4
ENPEP	Glutamyl Aminopeptidase
ZMPSTE24	Zinc Metallopeptidase STE24
AMBP	Alpha-1-Microglobulin/Bikunin Precursor
NPNT	Nephronectin
CDK4	Cyclin Dependent Kinase 4
PLAU	Plasminogen Activator, Urokinase
RARA	Retinoic Acid Receptor Alpha
MTHFR	Methylenetetrahydrofolate Reductase
VLDLR	Very Low Density Lipoprotein Receptor
CYP11B2	Cytochrome P450 Family 11 Subfamily B Member 2
EYA1	EYA Transcriptional Coactivator And Phosphatase 1
GPX3	Glutathione Peroxidase 3
LTBP1	Latent Transforming Growth Factor Beta Binding Protein 1
IGFBP1	Insulin Like Growth Factor Binding Protein 1
PTPRU	Protein Tyrosine Phosphatase, Receptor Type U
MAGI1	Membrane Associated Guanylate Kinase, WW And PDZ Domain Containing 1
RAP1GAP	RAP1 GTPase Activating Protein
NPHP4	Nephrocystin 4
PDGFB	Platelet Derived Growth Factor Subunit B
SLC12A1	Solute Carrier Family 12 Member 1
FBXW7	F-Box And WD Repeat Domain Containing 7
FABP1	Fatty Acid Binding Protein 1
THBD	Thrombomodulin
CLCF1	Cardiotrophin Like Cytokine Factor 1
CHKA	Choline Kinase Alpha
IFNA2	Interferon Alpha 2
ECT2	Epithelial Cell Transforming 2
COG2	Component Of Oligomeric Golgi Complex 2
PDSS2	Decaprenyl Diphosphate Synthase Subunit 2
FMN1	Formin 1
SDK1	Sidekick Cell Adhesion Molecule 1
MIR186	MicroRNA 186
MIR193A	MicroRNA 193a
MTOR	Mechanistic Target Of Rapamycin Kinase
HMGCR	3-Hydroxy-3-Methylglutaryl-CoA Reductase
MMP2	Matrix Metallopeptidase 2
TGFBR1	Transforming Growth Factor Beta Receptor 1
A2M	Alpha-2-Macroglobulin
TFAM	Transcription Factor A, Mitochondrial
NRF1	Nuclear Respiratory Factor 1
IGFBP2	Insulin Like Growth Factor Binding Protein 2
SMAD1	SMAD Family Member 1
IGF1R	Insulin Like Growth Factor 1 Receptor
IGF1	Insulin Like Growth Factor 1
IRS1	Insulin Receptor Substrate 1
SRC	SRC Proto-Oncogene, Non-Receptor Tyrosine Kinase
SLC2A1	Solute Carrier Family 2 Member 1
APOC1	Apolipoprotein C1
GAPDH	Glyceraldehyde-3-Phosphate Dehydrogenase
GIPR	Gastric Inhibitory Polypeptide Receptor
F2RL3	F2R Like Thrombin Or Trypsin Receptor 3
DGKQ	Diacylglycerol Kinase Theta
VEGFA	Vascular Endothelial Growth Factor A
TIMP1	TIMP Metallopeptidase Inhibitor 1
RHOA	Ras Homolog Family Member A
MIF	Macrophage Migration Inhibitory Factor
IL4	Interleukin 4
MAPK14	Mitogen-Activated Protein Kinase 14
DDIT3	DNA Damage Inducible Transcript 3
RBP4	Retinol Binding Protein 4
SP1	Sp1 Transcription Factor
FOS	Fos Proto-Oncogene, AP-1 Transcription Factor Subunit
LDLR	Low Density Lipoprotein Receptor
TNFSF11	TNF Superfamily Member 11
SOD1	Superoxide Dismutase 1
TTC21B	Tetratricopeptide Repeat Domain 21B
RAC1	Rac Family Small GTPase 1
ANGPTL4	Angiopoietin Like 4
SMAD7	SMAD Family Member 7
MAPK1	Mitogen-Activated Protein Kinase 1
MPO	Myeloperoxidase
ACE2	Angiotensin I Converting Enzyme 2
MYC	MYC Proto-Oncogene, BHLH Transcription Factor
ABCB1	ATP Binding Cassette Subfamily B Member 1
HGF	Hepatocyte Growth Factor
B2M	Beta-2-Microglobulin
MAPK3	Mitogen-Activated Protein Kinase 3
ENG	Endoglin
PPARA	Peroxisome Proliferator Activated Receptor Alpha
BCL2	BCL2, Apoptosis Regulator
HMOX1	Heme Oxygenase 1
CCL5	C-C Motif Chemokine Ligand 5
IL15	Interleukin 15
HPX	Hemopexin
ESR1	Estrogen Receptor 1
EGF	Epidermal Growth Factor
CASP3	Caspase 3
NR3C1	Nuclear Receptor Subfamily 3 Group C Member 1
NRP1	Neuropilin 1
TNFRSF11A	TNF Receptor Superfamily Member 11a
CD2	CD2 Molecule
GREM1	Gremlin 1, DAN Family BMP Antagonist
MIR30A	MicroRNA 30a
CXCR4	C-X-C Motif Chemokine Receptor 4
JAK3	Janus Kinase 3
TLR3	Toll Like Receptor 3
FTH1	Ferritin Heavy Chain 1
NOTCH2	Notch 2
SIRT1	Sirtuin 1
EPAS1	Endothelial PAS Domain Protein 1
GGT1	Gamma-Glutamyltransferase 1
ABCA1	ATP Binding Cassette Subfamily A Member 1
CASP9	Caspase 9
NFATC1	Nuclear Factor Of Activated T Cells 1
YAP1	Yes Associated Protein 1
GFER	Growth Factor, Augmenter Of Liver Regeneration
CEBPA	CCAAT Enhancer Binding Protein Alpha
LIPC	Lipase C, Hepatic Type
HSP90B1	Heat Shock Protein 90 Beta Family Member 1
SMAD6	SMAD Family Member 6
ATF3	Activating Transcription Factor 3
PROM1	Prominin 1
AGTR2	Angiotensin II Receptor Type 2
LGALS1	Galectin 1
NRP2	Neuropilin 2
SP3	Sp3 Transcription Factor
DDN	Dendrin
CD24	CD24 Molecule
MIR30D	MicroRNA 30d
MET	MET Proto-Oncogene, Receptor Tyrosine Kinase
PRKCD	Protein Kinase C Delta
CTSD	Cathepsin D
CASP8	Caspase 8
FAS	Fas Cell Surface Death Receptor
TF	Transferrin
ALOX5	Arachidonate 5-Lipoxygenase
KRT18	Keratin 18
RELA	RELA Proto-Oncogene, NF-KB Subunit
BDNF	Brain Derived Neurotrophic Factor
CTLA4	Cytotoxic T-Lymphocyte Associated Protein 4
LTA4H	Leukotriene A4 Hydrolase
NLRP3	NLR Family Pyrin Domain Containing 3
HSPA5	Heat Shock Protein Family A (Hsp70) Member 5
HSPG2	Heparan Sulfate Proteoglycan 2
CXCL12	C-X-C Motif Chemokine Ligand 12
SPP1	Secreted Phosphoprotein 1
TRPV5	Transient Receptor Potential Cation Channel Subfamily V Member 5
COL4A6	Collagen Type IV Alpha 6 Chain
PDGFD	Platelet Derived Growth Factor D
IL13	Interleukin 13
IL9	Interleukin 9
HBEGF	Heparin Binding EGF Like Growth Factor
LTC4S	Leukotriene C4 Synthase
TRAF1	TNF Receptor Associated Factor 1
WWC1	WW And C2 Domain Containing 1
VASP	Vasodilator Stimulated Phosphoprotein
EPO	Erythropoietin
HHIP	Hedgehog Interacting Protein
GNPTAB	N-Acetylglucosamine-1-Phosphate Transferase Subunits Alpha And Beta
ADAM19	ADAM Metallopeptidase Domain 19
CAPZA1	Capping Actin Protein Of Muscle Z-Line Subunit Alpha 1
ATL1	Atlastin GTPase 1
PFN2	Profilin 2
PDLIM1	PDZ And LIM Domain 1
STK16	Serine/Threonine Kinase 16
IL7	Interleukin 7
TRPC1	Transient Receptor Potential Cation Channel Subfamily C Member 1
SNX9	Sorting Nexin 9
UBD	Ubiquitin D
EPB41L5	Erythrocyte Membrane Protein Band 4.1 Like 5
PDLIM2	PDZ And LIM Domain 2
ETV7	ETS Variant 7
ACTL7A	Actin Like 7A
MIR10A	MicroRNA 10a
MIR135A1	MicroRNA 135a-1
MIR135B	MicroRNA 135b
MIR217	MicroRNA 217
MIR378A	MicroRNA 378a
MIR135A2	MicroRNA 135a-2
MT-TL1	Mitochondrially Encoded TRNA Leucine 1 (UUA/G)
HNP1	Hypertensive Nephropathy
AGER	Advanced Glycosylation End-Product Specific Receptor
GLA	Galactosidase Alpha
CXCL8	C-X-C Motif Chemokine Ligand 8
AKR1B1	Aldo-Keto Reductase Family 1 Member B
JUN	Jun Proto-Oncogene, AP-1 Transcription Factor Subunit
NOS3	Nitric Oxide Synthase 3
COL4A2	Collagen Type IV Alpha 2 Chain
KNG1	Kininogen 1
MMP9	Matrix Metallopeptidase 9
TGFBR2	Transforming Growth Factor Beta Receptor 2
DES	Desmin
PRKCB	Protein Kinase C Beta
DCN	Decorin
VCAM1	Vascular Cell Adhesion Molecule 1
HRAS	HRas Proto-Oncogene, GTPase
CASP1	Caspase 1
IFNGR1	Interferon Gamma Receptor 1
NR1H2	Nuclear Receptor Subfamily 1 Group H Member 2
CFB	Complement Factor B
ANTXR2	ANTXR Cell Adhesion Molecule 2
MSR1	Macrophage Scavenger Receptor 1
CASP4	Caspase 4
HLA-DRB1	Major Histocompatibility Complex, Class II, DR Beta 1
IL12A	Interleukin 12A
COX5A	Cytochrome *C* Oxidase Subunit 5A
HP	Haptoglobin
PRTN3	Proteinase 3
OLR1	Oxidized Low Density Lipoprotein Receptor 1
HLA-DQB1	Major Histocompatibility Complex, Class II, DQ Beta 1
EREG	Epiregulin
DIAPH2	Diaphanous Related Formin 2
AZGP1	Alpha-2-Glycoprotein 1, Zinc-Binding
AREG	Amphiregulin
PTAFR	Platelet Activating Factor Receptor
TLE4	Transducin Like Enhancer Of Split 4
IL12B	Interleukin 12B
BPI	Bactericidal Permeability Increasing Protein
SCGB1A1	Secretoglobin Family 1A Member 1
IFNA1	Interferon Alpha 1
SEMA4C	Semaphorin 4C
ADCK2	AarF Domain Containing Kinase 2
MIR196A2	MicroRNA 196a-2
MIR490	MicroRNA 490
SMAD4	SMAD Family Member 4
EDNRA	Endothelin Receptor Type A
PLAT	Plasminogen Activator, Tissue Type
E2F1	E2F Transcription Factor 1
ITIH4	Inter-Alpha-Trypsin Inhibitor Heavy Chain Family Member 4
MIR21	MicroRNA 21
MMP1	Matrix Metallopeptidase 1
CAT	Catalase
MAPK10	Mitogen-Activated Protein Kinase 10
PARP1	Poly(ADP-Ribose) Polymerase 1
RB1	RB Transcriptional Corepressor 1
ESR2	Estrogen Receptor 2
CD36	CD36 Molecule
GDNF	Glial Cell Derived Neurotrophic Factor
LEP	Leptin
NPPA	Natriuretic Peptide A
MBL2	Mannose Binding Lectin 2
CST3	Cystatin C
SEMA3A	Semaphorin 3A
THBS1	Thrombospondin 1
UMOD	Uromodulin
SERPINB7	Serpin Family B Member 7
AKT2	AKT Serine/Threonine Kinase 2
NFKB1	Nuclear Factor Kappa B Subunit 1
STAT3	Signal Transducer And Activator Of Transcription 3
CDC42	Cell Division Cycle 42
CYP3A4	Cytochrome P450 Family 3 Subfamily A Member 4
NFKBIA	NFKB Inhibitor Alpha
MAPK8	Mitogen-Activated Protein Kinase 8
CD40	CD40 Molecule
C3	Complement C3
PLG	Plasminogen
MMP7	Matrix Metallopeptidase 7
PTK2B	Protein Tyrosine Kinase 2 Beta
DDX58	DExD/H-Box Helicase 58
COL4A1	Collagen Type IV Alpha 1 Chain
PIK3CG	Phosphatidylinositol-4,5-Bisphosphate 3-Kinase Catalytic Subunit Gamma
MYH7	Myosin Heavy Chain 7
IGF2	Insulin Like Growth Factor 2
ECE1	Endothelin Converting Enzyme 1
C5	Complement C5
COL1A2	Collagen Type I Alpha 2 Chain
PROS1	Protein S
MYH6	Myosin Heavy Chain 6
TNC	Tenascin C
VCAN	Versican
GFPT1	Glutamine–Fructose-6-Phosphate Transaminase 1
EDN3	Endothelin 3
CCR1	C-C Motif Chemokine Receptor 1
ADIPOQ	Adiponectin, C1Q And Collagen Domain Containing
TRIO	Trio Rho Guanine Nucleotide Exchange Factor
FABP4	Fatty Acid Binding Protein 4
CCR2	C-C Motif Chemokine Receptor 2
CSF1	Colony Stimulating Factor 1
BMP7	Bone Morphogenetic Protein 7
S100A8	S100 Calcium Binding Protein A8
MLXIPL	MLX Interacting Protein Like
TNFRSF12A	TNF Receptor Superfamily Member 12A
PLTP	Phospholipid Transfer Protein
PDPN	Podoplanin
NID1	Nidogen 1
FMOD	Fibromodulin
NES	Nestin
SLC25A17	Solute Carrier Family 25 Member 17
TNFSF12	TNF Superfamily Member 12
USF2	Upstream Transcription Factor 2, C-Fos Interacting
ZFYVE9	Zinc Finger FYVE-Type Containing 9
PITRM1	Pitrilysin Metallopeptidase 1
SMPDL3B	Sphingomyelin Phosphodiesterase Acid Like 3B
CCN1	Cellular Communication Network Factor 1
PDGFRA	Platelet Derived Growth Factor Receptor Alpha
EGFR	Epidermal Growth Factor Receptor
PDGFRB	Platelet Derived Growth Factor Receptor Beta
JAK2	Janus Kinase 2
KDR	Kinase Insert Domain Receptor
MAP2K1	Mitogen-Activated Protein Kinase Kinase 1
MAP2K2	Mitogen-Activated Protein Kinase Kinase 2
INSR	Insulin Receptor
AR	Androgen Receptor
AKT3	AKT Serine/Threonine Kinase 3
PIK3CA	Phosphatidylinositol-4,5-Bisphosphate 3-Kinase Catalytic Subunit Alpha
PTEN	Phosphatase And Tensin Homolog
STAT1	Signal Transducer And Activator Of Transcription 1
CDK5	Cyclin Dependent Kinase 5
ADK	Adenosine Kinase
MMP3	Matrix Metallopeptidase 3
UCHL1	Ubiquitin C-Terminal Hydrolase L1
CD4	CD4 Molecule
CDKN2A	Cyclin Dependent Kinase Inhibitor 2A
CTSB	Cathepsin B
CASP7	Caspase 7
ACVRL1	Activin A Receptor Like Type 1
ADAM17	ADAM Metallopeptidase Domain 17
PPIB	Peptidylprolyl Isomerase B
HSPB1	Heat Shock Protein Family B (Small) Member 1
YWHAE	Tyrosine 3-Monooxygenase/Tryptophan 5-Monooxygenase Activation Protein Epsilon
GATA3	GATA Binding Protein 3
JAK1	Janus Kinase 1
HDAC3	Histone Deacetylase 3
NTRK1	Neurotrophic Receptor Tyrosine Kinase 1
NOS1	Nitric Oxide Synthase 1
CCNE1	Cyclin E1
ACACA	Acetyl-CoA Carboxylase Alpha
CAV1	Caveolin 1
PRKCZ	Protein Kinase C Zeta
SGK1	Serum/Glucocorticoid Regulated Kinase 1
NR3C2	Nuclear Receptor Subfamily 3 Group C Member 2
SLC5A1	Solute Carrier Family 5 Member 1
TFRC	Transferrin Receptor
TGFB2	Transforming Growth Factor Beta 2
VWF	Von Willebrand Factor
FOXO1	Forkhead Box O1
CYP3A5	Cytochrome P450 Family 3 Subfamily A Member 5
FASLG	Fas Ligand
CCR5	C-C Motif Chemokine Receptor 5 (Gene/Pseudogene)
CES1	Carboxylesterase 1
CNR1	Cannabinoid Receptor 1
PPARD	Peroxisome Proliferator Activated Receptor Delta
SELP	Selectin P
MMP10	Matrix Metallopeptidase 10
NR1H3	Nuclear Receptor Subfamily 1 Group H Member 3
MS4A1	Membrane Spanning 4-Domains A1
SPHK1	Sphingosine Kinase 1
LRP1	LDL Receptor Related Protein 1
HDAC9	Histone Deacetylase 9
TGFA	Transforming Growth Factor Alpha
TRAF3	TNF Receptor Associated Factor 3
TRAF6	TNF Receptor Associated Factor 6
TSHR	Thyroid Stimulating Hormone Receptor
ADORA2B	Adenosine A2b Receptor
BID	BH3 Interacting Domain Death Agonist
CA8	Carbonic Anhydrase 8
CDK5R1	Cyclin Dependent Kinase 5 Regulatory Subunit 1
CFH	Complement Factor H
CDK1	Cyclin Dependent Kinase 1
ANXA5	Annexin A5
ANG	Angiogenin
ITGB6	Integrin Subunit Beta 6
LNPEP	Leucyl And Cystinyl Aminopeptidase
SERPINH1	Serpin Family H Member 1
S100B	S100 Calcium Binding Protein B
TBX3	T-Box 3
PXN	Paxillin
TGIF1	TGFB Induced Factor Homeobox 1
TNFSF13B	TNF Superfamily Member 13b
ZYX	Zyxin
GH1	Growth Hormone 1
CX3CR1	C-X3-C Motif Chemokine Receptor 1
LGALS3	Galectin 3
HIPK2	Homeodomain Interacting Protein Kinase 2
STMN1	Stathmin 1
HPSE	Heparanase
EGR1	Early Growth Response 1
CD34	CD34 Molecule
EEF1A1	Eukaryotic Translation Elongation Factor 1 Alpha 1
CTNS	Cystinosin, Lysosomal Cystine Transporter
BDKRB2	Bradykinin Receptor B2
HDAC7	Histone Deacetylase 7
IQGAP1	IQ Motif Containing GTPase Activating Protein 1
SALL1	Spalt Like Transcription Factor 1
MPZ	Myelin Protein Zero
MEFV	MEFV, Pyrin Innate Immunity Regulator
TAT	Tyrosine Aminotransferase
SPI1	Spi-1 Proto-Oncogene
RAB3A	RAB3A, Member RAS Oncogene Family
USF1	Upstream Transcription Factor 1
FOXO3	Forkhead Box O3
DDAH2	Dimethylarginine Dimethylaminohydrolase 2
FCGR3B	Fc Fragment Of IgG Receptor IIIb
IL17A	Interleukin 17A
P2RX4	Purinergic Receptor P2X 4
PLXNA1	Plexin A1
TG	Thyroglobulin
TNFRSF6B	TNF Receptor Superfamily Member 6b
CSRP3	Cysteine And Glycine Rich Protein 3
ACTC1	Actin, Alpha, Cardiac Muscle 1
C4A	Complement C4A (Rodgers Blood Group)
TAGLN	Transgelin
ID1	Inhibitor Of DNA Binding 1, HLH Protein
CCL4	C-C Motif Chemokine Ligand 4
FCAR	Fc Fragment Of IgA Receptor
CAMP	Cathelicidin Antimicrobial Peptide
COL8A2	Collagen Type VIII Alpha 2 Chain
ST3GAL4	ST3 Beta-Galactoside Alpha-2,3-Sialyltransferase 4
IL1RL1	Interleukin 1 Receptor Like 1
WASL	Wiskott-Aldrich Syndrome Like
CHIA	Chitinase, Acidic
BPHL	Biphenyl Hydrolase Like
KLF15	Kruppel Like Factor 15
PLA2R1	Phospholipase A2 Receptor 1
RHOD	Ras Homolog Family Member D
SCAP	SREBF Chaperone
PDLIM5	PDZ And LIM Domain 5
RPH3A	Rabphilin 3A
HIST1H1B	Histone Cluster 1 H1 Family Member B
CCL3	C-C Motif Chemokine Ligand 3
COL8A1	Collagen Type VIII Alpha 1 Chain
PECAM1	Platelet And Endothelial Cell Adhesion Molecule 1
P3H1	Prolyl 3-Hydroxylase 1
NUP133	Nucleoporin 133
SNF8	SNF8, ESCRT-II Complex Subunit
TSLP	Thymic Stromal Lymphopoietin
ACTN3	Actinin Alpha 3 (Gene/Pseudogene)
LECT2	Leukocyte Cell Derived Chemotaxin 2
WDR19	WD Repeat Domain 19
CSN1S1	Casein Alpha S1
GOLIM4	Golgi Integral Membrane Protein 4
MPV17L	MPV17 Mitochondrial Inner Membrane Protein Like
WTIP	WT1 Interacting Protein
HIST2H3C	Histone Cluster 2 H3 Family Member C
KRBOX4	KRAB Box Domain Containing 4
MIR216A	MicroRNA 216a
MBL3P	Mannose-Binding Lectin Family Member 3, Pseudogene

**Table 3:** Information for target genes of tripterygium from TCMSP database

Mol Id	Gene Name	Mol name
MOL000296	PGR	hederagenin
MOL000296	NCOA2	hederagenin
MOL000296	CHRM3	hederagenin
MOL000296	CHRM1	hederagenin
MOL000296	CHRM2	hederagenin
MOL000296	ADRA1B	hederagenin
MOL000296	GABRA1	hederagenin
MOL000296	GRIA2	hederagenin
MOL000296	ADH1B	hederagenin
MOL000296	ADH1C	hederagenin
MOL000296	LYZ	hederagenin
MOL000296	PTGS1	hederagenin
MOL000296	SCN5A	hederagenin
MOL000296	PTGS2	hederagenin
MOL000296	RXRA	hederagenin
MOL000296	SLC6A2	hederagenin
MOL003182	KCNH2	(+)-Medioresinol di-O-beta-D-glucopyranoside_qt
MOL003182	SCN5A	(+)-Medioresinol di-O-beta-D-glucopyranoside_qt
MOL003182	PTGS2	(+)-Medioresinol di-O-beta-D-glucopyranoside_qt
MOL003182	F7	(+)-Medioresinol di-O-beta-D-glucopyranoside_qt
MOL003184	PTGS1	81827-74-9
MOL003184	CHRM3	81827-74-9
MOL003184	KCNH2	81827-74-9
MOL003184	CHRM1	81827-74-9
MOL003184	SCN5A	81827-74-9
MOL003184	CHRM5	81827-74-9
MOL003184	PTGS2	81827-74-9
MOL003184	CHRM4	81827-74-9
MOL003184	OPRD1	81827-74-9
MOL003184	PGR	81827-74-9
MOL003184	CHRM2	81827-74-9
MOL003184	ADRA1B	81827-74-9
MOL003184	ADRB2	81827-74-9
MOL003184	OPRM1	81827-74-9
MOL003184	NCOA2	81827-74-9
MOL003184	NCOA1	81827-74-9
MOL003185	CHRM3	(1R,4aR,10aS)-5-hydroxy-1-(hydroxymethyl)-7-isopropyl-8-methoxy-1,4a -dimethyl-4,9,10,10a-tetrahydro-3H-phenanthren-2-one
MOL003185	CHRM1	(1R,4aR,10aS)-5-hydroxy-1-(hydroxymethyl)-7-isopropyl-8-methoxy-1,4a-dimethyl -4,9,10,10a-tetrahydro-3H-phenanthren-2-one
MOL003185	PTGS2	(1R,4aR,10aS)-5-hydroxy-1-(hydroxymethyl)-7-isopropyl-8-methoxy-1,4a-dimethyl -4,9,10,10a-tetrahydro-3H-phenanthren-2-one
MOL003185	OPRD1	(1R,4aR,10aS)-5-hydroxy-1-(hydroxymethyl)-7-isopropyl-8-methoxy-1,4a-dimethyl -4,9,10,10a-tetrahydro-3H-phenanthren-2-one
MOL003185	ADRA1A	(1R,4aR,10aS)-5-hydroxy-1-(hydroxymethyl)-7-isopropyl-8-methoxy-1,4a-dimethyl- 4,9,10,10a-tetrahydro-3H-phenanthren-2-one
MOL003185	ADRA1B	(1R,4aR,10aS)-5-hydroxy-1-(hydroxymethyl)-7-isopropyl-8-methoxy-1,4a-dimethyl- 4,9,10,10a-tetrahydro-3H-phenanthren-2-one
MOL003185	ADRA1D	(1R,4aR,10aS)-5-hydroxy-1-(hydroxymethyl)-7-isopropyl-8-methoxy-1,4a-dimethyl- 4,9,10,10a-tetrahydro-3H-phenanthren-2-one
MOL003185	OPRM1	(1R,4aR,10aS)-5-hydroxy-1-(hydroxymethyl)-7-isopropyl-8-methoxy-1,4a-dimethyl- 4,9,10,10a-tetrahydro-3H-phenanthren-2-one
MOL003185	NR3C1	(1R,4aR,10aS)-5-hydroxy-1-(hydroxymethyl)-7-isopropyl-8-methoxy-1,4a-dimethyl- 4,9,10,10a-tetrahydro-3H-phenanthren-2-one
MOL003185	NCOA2	(1R,4aR,10aS)-5-hydroxy-1-(hydroxymethyl)-7-isopropyl-8-methoxy-1,4a-dimethyl- 4,9,10,10a-tetrahydro-3H-phenanthren-2-one
MOL003185	NCOA1	(1R,4aR,10aS)-5-hydroxy-1-(hydroxymethyl)-7-isopropyl-8-methoxy-1,4a-dimethyl- 4,9,10,10a-tetrahydro-3H-phenanthren-2-one
MOL003185	SCN5A	(1R,4aR,10aS)-5-hydroxy-1-(hydroxymethyl)-7-isopropyl-8-methoxy-1,4a-dimethyl- 4,9,10,10a-tetrahydro-3H-phenanthren-2-one
MOL003185	CHRM2	(1R,4aR,10aS)-5-hydroxy-1-(hydroxymethyl)-7-isopropyl-8-methoxy-1,4a-dimethyl- 4,9,10,10a-tetrahydro-3H-phenanthren-2-one
MOL003185	ADRB2	(1R,4aR,10aS)-5-hydroxy-1-(hydroxymethyl)-7-isopropyl-8-methoxy-1,4a-dimethyl- 4,9,10,10a-tetrahydro-3H-phenanthren-2-one
MOL003187	RELA	triptolide
MOL003187	STAT3	triptolide
MOL003187	VEGFA	triptolide
MOL003187	BCL2	triptolide
MOL003187	FOS	triptolide
MOL003187	CDKN1A	triptolide
MOL003187	PLAU	triptolide
MOL003187	TNFSF15	triptolide
MOL003187	JUN	triptolide
MOL003187	CASP3	triptolide
MOL003187	TP63	triptolide
MOL003187	MAPK8	triptolide
MOL003187	PTGS2	triptolide
MOL003187	STAT1	triptolide
MOL003187	CXCL8	triptolide
MOL003187	MCL1	triptolide
MOL003187	IL2	triptolide
MOL003187	IFNG	triptolide
MOL003187	IL4	triptolide
MOL003187	CD80	triptolide
MOL003187	CD86	triptolide
MOL003187	CXCR4	triptolide
MOL003187	BIRC3	triptolide
MOL003187	CD274	triptolide
MOL003187	IL23A	triptolide
MOL003187	CCR7	triptolide
MOL003187	CD1A	triptolide
MOL003187	CD40	triptolide
MOL003187	CD14	triptolide
MOL003187	C3	triptolide
MOL003187	VTCN1	triptolide
MOL003196	CHRM3	Tryptophenolide
MOL003196	KCNH2	Tryptophenolide
MOL003196	CHRM1	Tryptophenolide
MOL003196	SCN5A	Tryptophenolide
MOL003196	CHRM5	Tryptophenolide
MOL003196	PTGS2	Tryptophenolide
MOL003196	RXRA	Tryptophenolide
MOL003196	OPRD1	Tryptophenolide
MOL003196	ADRA1A	Tryptophenolide
MOL003196	PGR	Tryptophenolide
MOL003196	CHRM2	Tryptophenolide
MOL003196	ADRA1B	Tryptophenolide
MOL003196	ADRB2	Tryptophenolide
MOL003196	ADRA1D	Tryptophenolide
MOL003196	OPRM1	Tryptophenolide
MOL003196	NCOA2	Tryptophenolide
MOL003196	NCOA1	Tryptophenolide
MOL003199	NOS2	5,8-Dihydroxy-7-(4-hydroxy-5-methyl-coumarin-3)-coumarin
MOL003199	PTGS1	5,8-Dihydroxy-7-(4-hydroxy-5-methyl-coumarin-3)-coumarin
MOL003199	KCNH2	5,8-Dihydroxy-7-(4-hydroxy-5-methyl-coumarin-3)-coumarin
MOL003199	ESR1	5,8-Dihydroxy-7-(4-hydroxy-5-methyl-coumarin-3)-coumarin
MOL003199	AR	5,8-Dihydroxy-7-(4-hydroxy-5-methyl-coumarin-3)-coumarin
MOL003199	SCN5A	5,8-Dihydroxy-7-(4-hydroxy-5-methyl-coumarin-3)-coumarin
MOL003199	PPARG	5,8-Dihydroxy-7-(4-hydroxy-5-methyl-coumarin-3)-coumarin
MOL003199	PTGS2	5,8-Dihydroxy-7-(4-hydroxy-5-methyl-coumarin-3)-coumarin
MOL003199	F7	5,8-Dihydroxy-7-(4-hydroxy-5-methyl-coumarin-3)-coumarin
MOL003199	KDR	5,8-Dihydroxy-7-(4-hydroxy-5-methyl-coumarin-3)-coumarin
MOL003199	PYGM	5,8-Dihydroxy-7-(4-hydroxy-5-methyl-coumarin-3)-coumarin
MOL003199	PRSS1	5,8-Dihydroxy-7-(4-hydroxy-5-methyl-coumarin-3)-coumarin
MOL003209	KCNH2	Celallocinnine
MOL003209	SCN5A	Celallocinnine
MOL003217	NOS2	Isoxanthohumol
MOL003217	KCNH2	Isoxanthohumol
MOL003217	ESR1	Isoxanthohumol
MOL003217	SCN5A	Isoxanthohumol
MOL003217	PTGS2	Isoxanthohumol
MOL003217	KDR	Isoxanthohumol
MOL003217	ADRA1B	Isoxanthohumol
MOL003217	ADRB2	Isoxanthohumol
MOL003217	NCOA2	Isoxanthohumol
MOL003217	NCOA1	Isoxanthohumol
MOL003217	PTGS1	Isoxanthohumol
MOL003217	PPARD	Isoxanthohumol
MOL003224	NR3C2	Tripdiotolnide
MOL003225	NR3C2	Hypodiolide A
MOL003225	NR3C1	Hypodiolide A
MOL003229	CHRM3	Triptinin B
MOL003229	KCNH2	Triptinin B
MOL003229	CHRM1	Triptinin B
MOL003229	SCN5A	Triptinin B
MOL003229	CHRM5	Triptinin B
MOL003229	PTGS2	Triptinin B
MOL003229	RXRA	Triptinin B
MOL003229	ADRA1A	Triptinin B
MOL003229	PGR	Triptinin B
MOL003229	CHRM2	Triptinin B
MOL003229	ADRA1B	Triptinin B
MOL003229	ADRB2	Triptinin B
MOL003229	ADRA1D	Triptinin B
MOL003229	OPRM1	Triptinin B
MOL003229	NR3C1	Triptinin B
MOL003229	RXRB	Triptinin B
MOL003229	NCOA2	Triptinin B
MOL003229	NCOA1	Triptinin B
MOL003231	PTGS1	Triptoditerpenic acid B
MOL003231	CHRM3	Triptoditerpenic acid B
MOL003231	KCNH2	Triptoditerpenic acid B
MOL003231	CHRM1	Triptoditerpenic acid B
MOL003231	SCN5A	Triptoditerpenic acid B
MOL003231	CHRM5	Triptoditerpenic acid B
MOL003231	PTGS2	Triptoditerpenic acid B
MOL003231	CHRM4	Triptoditerpenic acid B
MOL003231	RXRA	Triptoditerpenic acid B
MOL003231	OPRD1	Triptoditerpenic acid B
MOL003231	ADRA1A	Triptoditerpenic acid B
MOL003231	PGR	Triptoditerpenic acid B
MOL003231	CHRM2	Triptoditerpenic acid B
MOL003231	ADRA1B	Triptoditerpenic acid B
MOL003231	ADRB2	Triptoditerpenic acid B
MOL003231	ADRA1D	Triptoditerpenic acid B
MOL003231	OPRM1	Triptoditerpenic acid B
MOL003231	NR3C1	Triptoditerpenic acid B
MOL003231	RXRB	Triptoditerpenic acid B
MOL003231	NCOA2	Triptoditerpenic acid B
MOL003231	NCOA1	Triptoditerpenic acid B
MOL003245	CHRM3	Triptonoditerpenic acid
MOL003245	KCNH2	Triptonoditerpenic acid
MOL003245	CHRM1	Triptonoditerpenic acid
MOL003245	SCN5A	Triptonoditerpenic acid
MOL003245	PTGS2	Triptonoditerpenic acid
MOL003245	OPRD1	Triptonoditerpenic acid
MOL003245	ADRA1B	Triptonoditerpenic acid
MOL003245	ADRB2	Triptonoditerpenic acid
MOL003245	NCOA2	Triptonoditerpenic acid
MOL003245	NCOA1	Triptonoditerpenic acid
MOL003248	PTGS1	Triptonoterpene
MOL003248	CHRM3	Triptonoterpene
MOL003248	CHRM1	Triptonoterpene
MOL003248	SCN5A	Triptonoterpene
MOL003248	PTGS2	Triptonoterpene
MOL003248	RXRA	Triptonoterpene
MOL003248	ACHE	Triptonoterpene
MOL003248	ADRA1A	Triptonoterpene
MOL003248	PGR	Triptonoterpene
MOL003248	CHRM2	Triptonoterpene
MOL003248	ADRA1B	Triptonoterpene
MOL003248	ADRB2	Triptonoterpene
MOL003248	ADRA1D	Triptonoterpene
MOL003248	OPRM1	Triptonoterpene
MOL003248	NR3C1	Triptonoterpene
MOL003248	NCOA2	Triptonoterpene
MOL003248	NCOA1	Triptonoterpene
MOL003266	PGR	21-Hydroxy-30-norhopan-22-one
MOL003280	CHRM3	TRIPTONOLIDE
MOL003280	CHRM1	TRIPTONOLIDE
MOL003280	SCN5A	TRIPTONOLIDE
MOL003280	CHRM5	TRIPTONOLIDE
MOL003280	PTGS2	TRIPTONOLIDE
MOL003280	OPRD1	TRIPTONOLIDE
MOL003280	ADRA1A	TRIPTONOLIDE
MOL003280	PGR	TRIPTONOLIDE
MOL003280	CHRM2	TRIPTONOLIDE
MOL003280	ADRB2	TRIPTONOLIDE
MOL003280	OPRM1	TRIPTONOLIDE
MOL003280	NCOA2	TRIPTONOLIDE
MOL003280	NCOA1	TRIPTONOLIDE
MOL000358	PGR	beta-sitosterol
MOL000358	NCOA2	beta-sitosterol
MOL000358	PTGS1	beta-sitosterol
MOL000358	PTGS2	beta-sitosterol
MOL000358	KCNH2	beta-sitosterol
MOL000358	CHRM3	beta-sitosterol
MOL000358	CHRM1	beta-sitosterol
MOL000358	SCN5A	beta-sitosterol
MOL000358	CHRM4	beta-sitosterol
MOL000358	ADRA1A	beta-sitosterol
MOL000358	CHRM2	beta-sitosterol
MOL000358	ADRA1B	beta-sitosterol
MOL000358	ADRB2	beta-sitosterol
MOL000358	CHRNA2	beta-sitosterol
MOL000358	SLC6A4	beta-sitosterol
MOL000358	OPRM1	beta-sitosterol
MOL000358	GABRA1	beta-sitosterol
MOL000358	BCL2	beta-sitosterol
MOL000358	BAX	beta-sitosterol
MOL000358	CASP9	beta-sitosterol
MOL000358	JUN	beta-sitosterol
MOL000358	CASP3	beta-sitosterol
MOL000358	CASP8	beta-sitosterol
MOL000358	PRKCA	beta-sitosterol
MOL000358	PON1	beta-sitosterol
MOL000358	MAP2	beta-sitosterol
MOL000211	PGR	Mairin
MOL000422	NOS2	kaempferol
MOL000422	PTGS1	kaempferol
MOL000422	AR	kaempferol
MOL000422	PPARG	kaempferol
MOL000422	PTGS2	kaempferol
MOL000422	NCOA2	kaempferol
MOL000422	PRSS1	kaempferol
MOL000422	PGR	kaempferol
MOL000422	CHRM1	kaempferol
MOL000422	ACHE	kaempferol
MOL000422	SLC6A2	kaempferol
MOL000422	CHRM2	kaempferol
MOL000422	ADRA1B	kaempferol
MOL000422	GABRA1	kaempferol
MOL000422	F7	kaempferol
MOL000422	RELA	kaempferol
MOL000422	IKBKB	kaempferol
MOL000422	AKT1	kaempferol
MOL000422	BCL2	kaempferol
MOL000422	BAX	kaempferol
MOL000422	TNFSF15	kaempferol
MOL000422	JUN	kaempferol
MOL000422	AHSA1	kaempferol
MOL000422	CASP3	kaempferol
MOL000422	MAPK8	kaempferol
MOL000422	MMP1	kaempferol
MOL000422	STAT1	kaempferol
MOL000422	PPARG	kaempferol
MOL000422	HMOX1	kaempferol
MOL000422	CYP3A4	kaempferol
MOL000422	CYP1A2	kaempferol
MOL000422	CYP1A1	kaempferol
MOL000422	ICAM1	kaempferol
MOL000422	SELE	kaempferol
MOL000422	VCAM1	kaempferol
MOL000422	NR1I2	kaempferol
MOL000422	CYP1B1	kaempferol
MOL000422	ALOX5	kaempferol
MOL000422	HAS2	kaempferol
MOL000422	GSTP1	kaempferol
MOL000422	AHR	kaempferol
MOL000422	PSMD3	kaempferol
MOL000422	SLC2A4	kaempferol
MOL000422	NR1I3	kaempferol
MOL000422	INSR	kaempferol
MOL000422	DIO1	kaempferol
MOL000422	PPP3CA	kaempferol
MOL000422	GSTM1	kaempferol
MOL000422	GSTM2	kaempferol
MOL000422	AKR1C3	kaempferol
MOL000422	SLPI	kaempferol
MOL000449	PGR	Stigmasterol
MOL000449	NR3C2	Stigmasterol
MOL000449	NCOA2	Stigmasterol
MOL000449	ADH1C	Stigmasterol
MOL000449	RXRA	Stigmasterol
MOL000449	NCOA1	Stigmasterol
MOL000449	PTGS1	Stigmasterol
MOL000449	PTGS2	Stigmasterol
MOL000449	ADRA2A	Stigmasterol
MOL000449	SLC6A2	Stigmasterol
MOL000449	SLC6A3	Stigmasterol
MOL000449	ADRB2	Stigmasterol
MOL000449	AKR1B1	Stigmasterol
MOL000449	PLAU	Stigmasterol
MOL000449	LTA4H	Stigmasterol
MOL000449	MAOB	Stigmasterol
MOL000449	MAOA	Stigmasterol
MOL000449	CTRB1	Stigmasterol
MOL000449	CHRM3	Stigmasterol
MOL000449	CHRM1	Stigmasterol
MOL000449	ADRB1	Stigmasterol
MOL000449	SCN5A	Stigmasterol
MOL000449	ADRA1A	Stigmasterol
MOL000449	CHRM2	Stigmasterol
MOL000449	ADRA1B	Stigmasterol
MOL000449	GABRA1	Stigmasterol
MOL002058	KCNH2	40957-99-1
MOL002058	SCN5A	40957-99-1
MOL002058	PTGS2	40957-99-1
MOL002058	PTGS1	40957-99-1
MOL002058	NCOA2	40957-99-1
MOL002058	F7	40957-99-1
MOL003283	ESR1	(2R,3R,4S)-4-(4-hydroxy-3-methoxy-phenyl)-7-methoxy-2,3-dimethylol-tetralin-6-ol
MOL003283	AR	(2R,3R,4S)-4-(4-hydroxy-3-methoxy-phenyl)-7-methoxy-2,3-dimethylol-tetralin-6-ol
MOL003283	PPARG	(2R,3R,4S)-4-(4-hydroxy-3-methoxy-phenyl)-7-methoxy-2,3-dimethylol-tetralin-6-ol
MOL003283	PTGS2	(2R,3R,4S)-4-(4-hydroxy-3-methoxy-phenyl)-7-methoxy-2,3-dimethylol-tetralin-6-ol
MOL003283	F7	(2R,3R,4S)-4-(4-hydroxy-3-methoxy-phenyl)-7-methoxy-2,3-dimethylol-tetralin-6-ol
MOL003283	ADRB2	(2R,3R,4S)-4-(4-hydroxy-3-methoxy-phenyl)-7-methoxy-2,3-dimethylol-tetralin-6-ol
MOL003283	ESR2	(2R,3R,4S)-4-(4-hydroxy-3-methoxy-phenyl)-7-methoxy-2,3-dimethylol-tetralin-6-ol
MOL003283	MAPK14	(2R,3R,4S)-4-(4-hydroxy-3-methoxy-phenyl)-7-methoxy-2,3-dimethylol-tetralin-6-ol
MOL003283	GSK3B	(2R,3R,4S)-4-(4-hydroxy-3-methoxy-phenyl)-7-methoxy-2,3-dimethylol-tetralin-6-ol
MOL003283	CHEK1	(2R,3R,4S)-4-(4-hydroxy-3-methoxy-phenyl)-7-methoxy-2,3-dimethylol-tetralin-6-ol
MOL003283	NCOA2	(2R,3R,4S)-4-(4-hydroxy-3-methoxy-phenyl)-7-methoxy-2,3-dimethylol-tetralin-6-ol
MOL003283	SCN5A	(2R,3R,4S)-4-(4-hydroxy-3-methoxy-phenyl)-7-methoxy-2,3-dimethylol-tetralin-6-ol
MOL003283	CCNA2	(2R,3R,4S)-4-(4-hydroxy-3-methoxy-phenyl)-7-methoxy-2,3-dimethylol-tetralin-6-ol
MOL003283	PTGS1	(2R,3R,4S)-4-(4-hydroxy-3-methoxy-phenyl)-7-methoxy-2,3-dimethylol-tetralin-6-ol
MOL004443	PTGS1	Zhebeiresinol
MOL004443	SCN5A	Zhebeiresinol
MOL004443	PTGS2	Zhebeiresinol
MOL004443	RXRA	Zhebeiresinol
MOL004443	ADRB2	Zhebeiresinol
MOL004443	GABRA1	Zhebeiresinol
MOL005828	NOS2	nobiletin
MOL005828	PTGS1	nobiletin
MOL005828	KCNH2	nobiletin
MOL005828	ESR1	nobiletin
MOL005828	AR	nobiletin
MOL005828	PPARG	nobiletin
MOL005828	PTGS2	nobiletin
MOL005828	F7	nobiletin
MOL005828	ESR2	nobiletin
MOL005828	CHEK1	nobiletin
MOL005828	PRSS1	nobiletin
MOL005828	NCOA2	nobiletin
MOL005828	GSK3B	nobiletin
MOL005828	SCN5A	nobiletin
MOL005828	BCL2	nobiletin
MOL005828	BAX	nobiletin
MOL005828	CASP9	nobiletin
MOL005828	MMP9	nobiletin
MOL005828	JUN	nobiletin
MOL005828	TP63	nobiletin
MOL005828	MAPK8	nobiletin
MOL005828	TIMP1	nobiletin
MOL005828	PPARG	nobiletin
MOL005828	CREB1	nobiletin
MOL005828	PLA2G4A	nobiletin
MOL005828	CD163	nobiletin
MOL005828	EPHB2	nobiletin
MOL007415	KCNH2	[(2S)-2-[[(2S)-2-(benzoylamino)-3-phenylpropanoyl]amino]-3-phenylpropyl] acetate
MOL007415	PTGS2	[(2S)-2-[[(2S)-2-(benzoylamino)-3-phenylpropanoyl]amino]-3-phenylpropyl] acetate
MOL007415	PRSS1	[(2S)-2-[[(2S)-2-(benzoylamino)-3-phenylpropanoyl]amino]-3-phenylpropyl] acetate
MOL007535	PGR	(5S,8S,9S,10R,13R,14S,17R)-17-[(1R,4R)-4-ethyl-1,5-dimethylhexyl]-10,13-dimethyl-2,4,5,7,8,9,11,12,14,15,16,17-dodecahydro-1H-cyclopenta[a]phenanthrene-3,6-dione
MOL009386	KCNH2	3,3′-bis-(3,4-dihydro-4-hydroxy-6-methoxy)-2H-1-benzopyran
MOL009386	ESR1	3,3′-bis-(3,4-dihydro-4-hydroxy-6-methoxy)-2H-1-benzopyran
MOL009386	PTGS2	3,3′-bis-(3,4-dihydro-4-hydroxy-6-methoxy)-2H-1-benzopyran
MOL009386	ADRB2	3,3′-bis-(3,4-dihydro-4-hydroxy-6-methoxy)-2H-1-benzopyran
MOL009386	CCNA2	3,3′-bis-(3,4-dihydro-4-hydroxy-6-methoxy)-2H-1-benzopyran

### Enrichment analysis of GO and KEGG

Forty-seven overlapping targets were screened for further investigation using the DAVID (htTPLs://david.ncifcrf.gov/) online tool. GO annotation results showed that the top 30 biological processes (BP) included cell apoptosis, proliferation of cells, positive signal transduction regulation, extracellular stimulus response, and cell death (Figure 2A). The results of KEGG enrichment analysis showed that the 47 overlapping targets were markedly enriched within 32 pathways, including the p53 signal transduction pathway, apoptosis, and the JAK-STAT signal transduction pathway (Figure 2B). *IL4* was mainly enriched in BP terms, including programmed cell death regulation, endogenous stimulus response, apoptosis regulation, positive cell proliferation regulation, and positive nitrogen compound metabolic process regulation. Based on the KEGG enrichment results, IL4 participated in the T-cell receptor signal transduction pathway, allograft rejection, intestinal IgA production immunologic network, the JAK-STAT signal transduction pathway, autoimmune thyroid disease, the Fc epsilon RI signal transduction pathway, and the interaction between cytokines and cytokine receptors.

**Figure 2:** Analysis of GO and KEGG Enrichment (**A**) 47 overlapped genes were analysis by GO annotation, which showed that the top 30 biological processes (BP). (**B**) 47 overlapped genes was analysis by KEGG, which enriched in 32 pathways.

### TPL alleviated kidney injury by inhibiting cell apoptosis in FSGS rats, and IL4 was up-regulated in kidney tissues of FSGS rats

FSGS rat models were established using external jugular vein cannulation; subsequently, the levels of BUN, 24-h urine protein, Scr, ALB, and TC were determined. Our results showed that the BUN, 24-h urine protein, TC, and Scr levels in FSGS animals were evidently decreased, while the ALB levels were significantly increased after the FSGS rats were administered TPL gavage (at 80 or 160 μg/(kg·d)) (Figure 3A–E). HE staining results showed that TPL significantly decreased the glomerulosclerosis index (GSI) in FSGS rats (Figure 3F,G). The apoptosis level was determined by TUNEL assay in the kidney tissues of FSGS rats. We found that FSGS promoted apoptosis in kidney tissues. However, TPL treatment suppressed the apoptosis of cells within the renal tissues of FSGS rats (Figure 4A,B). Therefore, we further detected the protein levels of IL4, nephrin, and podocin and the phosphorylation level of Stat6 using Western blotting. According to our results, TPL treatment decreased IL4 protein levels and stat6 activation, and increased the protein levels of nephrin and podocin in FSGS rats (Figure 4C–G).

**Figure 3:** TPL alleviated kidney injure in FSGS rats FSGS rat models were establised by using external jugular vein cannulation, (**A**) 24 h urine protein, (**B**) BUN, (**C**) Scr, (**D**) TC and (**E**) ALB levels were detected; (**F**) TPL could significantly decrease glomerulosclerosis index (GSI) of FSGS rats; (**G**) The pathomorphology of kidney in FSGS rats was showed by HE staining. Data are presented as the mean ± standard deviation. *^a^P*<0.05 versus Sham group, *^b^P*<0.05 versus FSGS group, and *^c^P*<0.05 versus TPL(80)+FSGS group.

**Figure 4:** TPL reduced cell apoptosis in FSGS rats FSGS rat models were established by using external jugular vein cannulation. (**A** and **B**) Apoptosis level was determined by TUNEL assay in kidney tissues of FSGS rats. (**C**) The protein levels of IL4, nephrin and podocin, and phosphorylation level of Stat6 by Western blotting analysis. (**D–G**) Histogram showed the statistical value. GAPDH was used as a load control. Data are presented as the mean ± standard deviation. *^a^P*<0.05 versus Sham group, *^b^P*<0.05 versus FSGS group, and *^c^P*<0.05 versus TPL(80)+FSGS group.

### TPL reversed the function of IL4 overexpression, promoting cell apoptosis

According to the results, 0–80 μmol/ml TPL had no influence on cell viability and apoptosis (Figure 5A–C). Western blotting results showed that 0–80 μmol/ml TPL minimally affected IL4, nephrin, and podocin expression and stat6 activation (Figure 5D). However, IL4 overexpression inhibited the viability and promoted apoptosis of podocytes. TPL inhibited IL4 overexpression-mediated cell apoptosis (Figure 6A–C). Furthermore, TPL decreased IL4 protein levels, increased nephrin and podocin protein levels, and inhibited the phosphorylation of Stat6 in podocytes (Figure 6D).

**Figure 5:** TPL has no influence on the cell viability and apoptosis (**A**) 0–80 μmol/ml of TPL little effected the viability of podocytes by CCK8 assay. (**B** and **C**) 0–80 μmol/ml of TPL little affected the apoptosis level of podocytes by flow cytometry assay. (**D**) The protein levels of IL4, nephrin and podocin, and phosphorylation level of Stat6 by Western blotting analysis. GAPDH was used as a load control. Data are presented as the mean ± standard deviation. *^a^P*<0.05 versus Sham group, *^b^P*<0.05 versus FSGS group, and *^c^P*<0.05 versus TPL(80)+FSGS group.

**Figure 6:** TPL reversed the function of IL4 overexpression promoting cell apoptosis (**A**) IL4 protein and mRNA levels were detected by Western blot and RT-PCR assays. (**B**) The viability of podocytes by CCK8 assay in cell with IL4. (**C**) The apoptosis level of podocytes by flow cytometry assay in cell with IL4. (**D**) The protein levels of nephrin and podocin, and phosphorylation level of Stat6 by Western blotting analysis. GAPDH was used as a load control. Data are presented as the mean ± standard deviation. *^a^P*<0.05 versus vector group, and *^b^P*<0.05 versus IL4 group.

## Discussion

The occurrence of FSGS is related to a variety of mechanisms. Podocyte injury is the central link of FSGS [16,17]. Glomerular sclerosis is the final pathological change in FSGS caused by the excessive accumulation of the glomerular extracellular matrix (ECM). Podocytes are an important part of the glomerulus and are the final barriers that block the filtration of plasma macromolecules. Apoptosis, fusion, and shedding of podocytes induced the occurrence and development of FSGS. TPL has been reported to have a protective effect on kidney damage [18]. Therefore, we constructed the Disease–Target–Compound network in the present study through the TCM network pharmacology to confirm the relationship between TPL and FSGS. It was further confirmed by constructing a PPT network that *IL4* was a target gene of TPL and FSGS. According to KEGG and GO enrichment analyses, *IL4* was closely related to apoptosis and was enriched in the JAK-STAT signal pathway. Thus, we proposed two hypotheses: (1) TPL can protect against FSGS kidney injury by inhibiting apoptosis; (2) The protective effect of TPL on FSGS-induced kidney damage may be achieved by targeting IL4.

IL-4 is an anti-inflammatory factor that belongs to the interleukin family [19]. It has been reported that IL4 can inhibit apoptosis of liver cancer cells, and blockage of the IL4/IL4R/STAT6 axis can promote apoptosis of Hodgkin lymphoma cells [20]. However, IL4 may also be involved in the disease as a pro-inflammatory factor [21]. The expression level of IL4 is high in kidney tissue with acute kidney injury [22]. Therefore, the effect of IL4 on FSGS should be more extensively investigated. IL4 activates stat6 by acting on the JAK-STAT signal pathway. Our results demonstrated that IL4 expression and the phosphorylation level of stat6 were up-regulated in kidney tissues of FSGS rats. This suggests that the IL/STAT6 signaling pathway is aberrantly activated in FSGS. TPL reduced apoptosis in the kidney tissue of FSGS rats while significantly inhibiting the expression of IL4 and the activation of stat6.

Nephrin and podocin are podocyte proteins that have been widely used to identify kidney injury [23,24]. It has been reported that podocin and nephrin levels were down-regulated in a kidney injury model to promote podocyte apoptosis, thereby aggravating kidney damage. Podocin and nephrin expression levels were remarkably down-regulated in the kidney tissue of FSGS rats. Similarly, TPL could upgrade the podocin and nephrin expression levels. This indicated that TPL attenuated glomerular sclerosis in FSGS rats by reducing podocyte apoptosis. To further investigate the mechanism of action of TPL on renal protection in FSGS rats, we carried out a study at the cellular level.

First, we need to investigate if 0–80 µmol/ml of TPL is toxic to podocyte. The functional experiment proved that TPL at low concentrations did not affect cell activity; cell apoptosis; the expression of IL4, nephrin, and podocin; and the activation of stat6, which excluded the threat of TPL for cells. The results showed that a high expression of IL4 inhibited cell viability, promoted apoptosis, increased phosphorylation of stat3, and inhibited the expression of nephrin and podocin. This suggested that a high expression of IL4 promoted apoptosis and aggravated glomerular sclerosis. TPL can reverse IL4-mediated podocyte apoptosis and reduce glomerular sclerosis.

In conclusion, up-regulation of IL4 in kidney tissue of FSGS rats activated stat6 and promoted podocyte apoptosis to aggravate glomerular sclerosis. TPL can alleviate glomerular sclerosis in FSGS rats by inhibiting the activation of the IL4/stat6 signaling pathway and podocyte apoptosis. This finding can offer a theoretical foundation for the application of TPL in treating FSGS.

## Data Availability

The datasets used and/or analyzed during the present study are available from the corresponding author on reasonable request.

## Abbreviations

FSGS: focal segmental glomerulosclerosis
GO: Gene Ontology
KEGG: Kyoto Encyclopedia of Genes and Genomes
PPI: protein–protein interaction
TCMSP: Traditional Chinese Medicine Systems Pharmacology Database
TPL: triptolide
